The article "Hsa-miR-623 suppresses tumor progression in human lung adenocarcinoma" was retracted in 2019. Reasons: contaminated cell lines or tissues; unreliable results or conclusions.

# Hsa-miR-623 suppresses tumor progression in human lung adenocarcinoma

**DOI:** 10.1038/cddis.2016.260

**Published:** 2016-09-29

**Authors:** Shuang Wei, Zun-yi Zhang, Sheng-ling Fu, Jun-gang Xie, Xian-sheng Liu, Yong-jian Xu, Jian-ping Zhao, Wei-ning Xiong

**Affiliations:** 1 Department of Respiratory and Critical Care Medicine, Key Laboratory of Pulmonary Diseases of Health Ministry, Key Cite of National Clinical Research Center for Respiratory Disease, Tongji Hospital, Tongji Medical College Huazhong University of Science and Technology, 1095 Jie Fang Avenue, Wuhan 430030, China; 2 Department of Surgery, Tongji Hospital, Tongji Medical College Huazhong University of Science and Technology, 1095 Jie Fang Da Dao, Wuhan 430030, China

## Abstract

Our previous study revealed that Ku80 was overexpressed in lung cancer tissues and hsa-miR-623 regulated the Ku80 expression; however, the detailed function of hsa-miR-623 in lung cancer was unclear. We identified that hsa-miR-623 bound to the 3'-UTR of Ku80 mRNA, thus significantly decreasing Ku80 expression in lung adenocarcinoma cells. Hsa-miR-623 was downregulated in lung adenocarcinoma tissues compared with corresponding non-tumorous tissues, and its expression was inversely correlated with Ku80 upregulation. Downregulation of hsa-miR-623 was associated with poor clinical outcomes of lung adenocarcinoma patients. Hsa-miR-623 suppressed lung adenocarcinoma cell proliferation, clonogenicity, migration and invasion *in vitro*. Hsa-miR-623 inhibited xenografts growth and metastasis of lung adenocarcinoma *in vivo*. Ku80 knockdown in lung adenocarcinoma cells suppressed tumor properties *in vitro* and *in vivo* similar to hsa-miR-623 overexpression. Further, hsa-miR-623 overexpression decreased matrix metalloproteinase-2 (MMP-2) and MMP-9 expression levels, with decreased ERK/JNK phosphorylation. Inhibition of hsa-miR-623 or overexpression of Ku80 promoted lung adenocarcinoma cell invasion, activated ERK/JNK phosphorylation and increased MMP-2/9 expressions, which could be reversed by ERK kinase inhibitor or JNK kinase inhibitor. In summary, our results showed that hsa-miR-623 was downregulated in lung adenocarcinoma and suppressed the invasion and metastasis targeting Ku80 through ERK/JNK inactivation mediated downregulation of MMP-2/9. These findings reveal that hsa-miR-623 may serve as an important therapeutic target in lung cancer therapy.

Lung cancer is the leading type of cancer-related deaths worldwide, likely because it is often diagnosed at advanced stages that are beyond the optimal treatment period.^1^ Non-small cell lung cancer (NSCLC) accounts for at least 80% of lung cancer cases, and these cases can be further categorized as adenocarcinoma (40%), squamous cell carcinoma (30–35%) and large cell carcinoma (5–15%).^1^ Despite advancements in treatments for NSCLC, the overall 5-year survival rate for NSCLC in the United States remains as low as 16% when considering all stages and subtypes.^2^ Lung cancers can develop a high metastatic potential, which is the major cause of treatment failure. The prognosis of patients with NSCLC principally correlates with tumor metastasis.^3^ More than 90% of lung cancer patients die of metastasis rather than from their primary tumors, suggesting that metastasis is a key prognostic factor.^4^ Therefore, further investigation of the molecular mechanisms underlying the metastasis of NSCLC is crucial for effective therapeutic targets.

The article "Hsa-miR-623 suppresses tumor progression in human lung adenocarcinoma" was retracted in 2019. Reasons: contaminated cell lines or tissues; unreliable results or conclusions.

Ku80 is well known for its critical function in repairing DNA double-strand breaks (DSBs).^5^ Misrepaired DSBs are major DNA lesions that can lead to chromosomal aberration, mutation or carcinogenesis.^6^ Previous studies have shown that overexpression of Ku80 may be associated with bladder cancer, cervical carcinoma, pancreatic cancer and gastric cancer.^7, 8, 9^ Our recent study observed that Ku80 was overexpressed in NSCLC tissues and Ku80 knockdown significantly suppressed NSCLC cell proliferation *in vitro* and *in vivo.*^10^ In another study, a significant overexpression of Ku80 was observed in primary human lung adenocarcinoma, which was associated with poor clinical outcomes and resistance to cisplatin-based chemotherapy.^11^ These studies provide evidence for a vital role of Ku80 in tumorigenesis. However, little is known about the role of Ku80 in tumor metastasis. In one study, a novel antibody (7B7) directed against the Ku70/Ku80 heterodimer was confirmed to block invasion in pancreatic and lung cancer cells.^12^ Ku80 was found to be involved in the migration process of thymosin beta4-regulated colon cancer cells.^13^ Thus, the relationship between Ku80 and cancer cell invasion needs further investigation. In addition, the molecular mechanisms underlying aberrant Ku80 expression and the precise role of Ku80 in the lung cancer invasion remain unexplored.

Metastatic potential of tumors depends in large part on the ability of the tumor to invade the extracellular matrix, a process that requires cells to lose intercellular adhesion molecules and to express proteolytic enzymes to facilitate invasion.^14^ Despite the fact that the search for detailed molecular mechanisms of NSCLC has been intensive, a number of questions concerning the basic nature of tumor metastasis remain incompletely understood.^14^ MicroRNAs (miRNAs) are a class of small noncoding RNAs that are approximately 22 nucleotides in length. MiRNAs can suppress post-transcriptional gene expression by binding to the 3′-untranslated regions (3′-UTRs) of mRNAs, effectively inhibiting translation or targeting mRNA degradation.^15, 16^ Studies have documented the role of miRNAs in the processes involved in tumor progression, including cellular proliferation, migration and invasion.^17, 18, 19^ The link between miRNAs and metastasis was first reported when miR-10b was shown to be involved in the promotion of breast cancer metastasis by direct targeting HOXD10.^20^ MicroRNA-145 was found to inhibit lung cancer cell metastasis.^21^ MicroRNA-135b promoted lung cancer metastasis by regulating multiple targets in the Hippo pathway and LZTS1.^22^ MicroRNA-33a inhibited lung cancer cell proliferation and invasion by regulating the expression of *β*-catenin.^23^ The novel miR-9500 repressed tumorigenesis and metastasis of human lung cancer by targeting the Akt1.^24^ MiR-125b was found to directly downregulate matrix metalloproteinase-13 (MMP-13) protein expression and inhibit the invasive capabilities of lung cancer cells.^25^ Taken together, these reports indicate that miRNAs are involved in the development and progression of tumor metastasis, and that miRNAs represent a potential target in the treatment of lung cancer. However, the roles of dysregulated miRNAs in lung cancer metastasis are still not fully elucidated. We successfully identified two miRNAs (hsa-miR-526b and hsa-miR-623) that could significantly inhibit Ku80 expression in A549 cells in our previous study.^10^ Our study had explored the function of hsa-miR-526b in NSCLC,^10^ so we chose to investigate the role of hsa-miR-623 in this paper.

The article "Hsa-miR-623 suppresses tumor progression in human lung adenocarcinoma" was retracted in 2019. Reasons: contaminated cell lines or tissues; unreliable results or conclusions.

The purpose of this study was to identify miRNAs that regulate Ku80 expression in lung cancer and determine their functions. We examined the expression patterns of miRNAs in lung adenocarcinoma tissues and evaluated the prognosis of patients with lung adenocarcinoma. To our knowledge, our data firstly revealed that hsa-miR-623 regulated lung adenocarcinoma cell growth, invasion and metastasis both *in vitro* and *in vivo* by directly targeting Ku80 genes. We also confirmed that the downregulation of MMP-2 and -9 through inactivating the ERK/JNK signaling pathway was involved in this process.

## Results

### Hsa-miR-623 directly targets Ku80 in lung adenocarcinoma cells

Previous studies^10^ indicated that Ku80 is overexpressed in lung adenocarcinoma tissues; however, molecular mechanisms have not been clear. To determine whether miRNAs were involved in regulating Ku80 expression, we applied the four most commonly used databases of miRNA to identify potential miRNAs that may target 3′-UTR of Ku80 mRNA. Nine miRNAs were consistently identified by these four miRNA databases (Supplementary Figure S1A). Upon this determination, we transiently transfected these miRNAs mimics into A549 cell lines and evaluated Ku80 expression levels using a western blot analysis. Among the nine miRNAs, the downregulation of Ku80 by the hsa-miR-526b and hsa-miR-623 mimics was the most pronounced (Supplementary Figure S1B). We have studied the effect of hsa-miR-526b on NSCLC cell proliferation in our previous study,^10^ thus we will further investigate the potential role of hsa-miR-623 in lung adenocarcinoma in this paper.

The article "Hsa-miR-623 suppresses tumor progression in human lung adenocarcinoma" was retracted in 2019. Reasons: contaminated cell lines or tissues; unreliable results or conclusions.

Subsequent luciferase assay indicated that hsa-miR-623 could directly target the binding site of wild-type 3′-UTR Ku80 mRNA and suppress luciferase expression of pLUC-Ku80 (*P*<0.01; Figures 1a and b). When the pLUC-mutant-Ku80 and miR-NC were examined in the similar manner, hsa-miR-623 failed to demonstrate this effect (*P*>0.05; Figure 1b). A549 and PC-9 cells were then treated with hsa-miR-623 mimics or inhibitors (Supplementary Figure S9). Overexpression of hsa-miR-623 mimics in A549 and PC-9 cell lines greatly reduced the protein level of Ku80 (*P*<0.05; Figure 1c). Conversely, inhibition of hsa-miR-623 increased Ku80 expression in both A549 and PC-9 cell lines (*P*<0.01; Figure 1d). Taken together, our data show that hsa-miR-623 negatively modulated Ku80 expression by directly binding to its 3′-UTR.

### Hsa-miR-623 is downregulated in lung adenocarcinoma tissues and its expression is associated with poor clinical outcomes

To further investigate its potential role, we evaluated the expression levels of hsa-miR-623 in 89 human lung adenocarcinoma tissues and their corresponding adjacent lung tissues using qRT-PCR. Interestingly, hsa-miR-623 was significantly downregulated in 80.9% lung adenocarcinoma tissues compared with adjacent lung tissues (*P*<0.0001 by paired *t*-test; Figure 2a). To further investigate whether the downregulated hsa-miR-623 is correlated with the lower survival rates of lung adenocarcinoma patients, we investigated a group of patients with lung adenocarcinoma. Kaplan–Meier log-rank analysis also indicated that lung adenocarcinoma patients with low hsa-miR-623 level had a significantly shorter median overall survival compared with those with high hsa-miR-623 expression (*P*=0.002; Figure 2b). Ku80 expression was examined in 89 cases of paired lung adenocarcinoma tissues and their corresponding adjacent lung tissues. A western blot analysis confirmed that Ku80 protein expression in 62 lung adenocarcinoma samples was higher compared with their adjacent lung tissues (*P*<0.0001; Figure 2c and Supplementary Figure S2). Kaplan–Meier log-rank analysis indicated that lung adenocarcinoma patients with high Ku80 level had a significantly shorter median overall survival compared with those with low Ku80 expression (Supplementary Figure S6). Moreover, the abundance of hsa-miR-623 was inversely correlated with that of Ku80 in lung adenocarcinoma tissues (*r*=−0.631, *P*<0.0001; Figure 2d). Next, we examined the correlation between hsa-miR-623 expression level and the clinicopathological parameters in patients with lung adenocarcinoma (shown in Supplementary Table S2). Hsa-miR-623 downregulation was significantly correlated with tumor differentiation, lymphatic metastasis and elevated serum carcinoembryonic antigen (CEA) level (*P*<0.05; Table 1). No correlation was found between miR-623 expression and other clinicopathological parameters in patients with lung adenocarcinoma (*P*>0.05; Table 1).

The article "Hsa-miR-623 suppresses tumor progression in human lung adenocarcinoma" was retracted in 2019. Reasons: contaminated cell lines or tissues; unreliable results or conclusions.

### Hsa-miR-623 suppresses the cell growth, migration and invasion of lung adenocarcinoma cells *in vitro*

The expression levels of hsa-miR-623 in A549 and PC-9 cells were significantly decreased compared with normal human bronchial epithelial (HBE) cells (*P*<0.05; Supplementary Figure S8). To investigate the effect of hsa-miR-623 on lung adenocarcinoma cell growth, hsa-miR-623-expressing lentiviral vector (GV252) and its negative control (NC) vector were transiently transfected into two lung adenocarcinoma cell lines, A549 and PC-9, respectively. Hsa-miR-623-expressing and NC-transfected stable A549 and PC-9 cell clones were generated. The qRT-PCR analysis confirmed that hsa-miR-623 stably expressing A549 cell clones (#1, #4 and #10) and PC-9 cell clones (#27, #28 and #29) expressed much higher levels of hsa-miR-623, whereas the clones with the NC showed very low level of hsa-miR-623 expression (*P*<0.05; Figure 3a). Western blot analysis also indicated that hsa-miR-623 stably expressing A549 and PC-9 cells expressed much lower protein levels of Ku80 than those of control cells (Supplementary Figure S3). Hsa-miR-623 overexpressing A549 and PC-9 stable clone cells grew at significantly slower rates compared with those of the NC-transfected cells (*P*<0.01; Figure 3b). Furthermore, to assess the functional role of hsa-miR-623 in tumor formation, the plate colony formation and anchorage-independent growth were measured in A549 and PC-9 cells. Analysis of clonogenicity showed that hsa-miR-623-overexpressing stable clone cells displayed much fewer and smaller colonies than NC-transfected cells (Supplementary Figure S4). Analysis of colony formation and cell growth showed that there was a significant difference among the different cell groups (*P*<0.05; Figures 3c and d).

The article "Hsa-miR-623 suppresses tumor progression in human lung adenocarcinoma" was retracted in 2019. Reasons: contaminated cell lines or tissues; unreliable results or conclusions.

To identify the role of hsa-miR-623 in lung adenocarcinoma metastasis, transwell insert chambers were introduced to investigate the impact of hsa-miR-623 on cell migration and invasion. The results showed that ectopic hsa-miR-623 expression significantly suppressed A549 and PC-9 cells migration and invasion as measured by crystal violet staining (*P*<0.05; Figures 3e–h).

Moreover, our further experiments indicated that miR-623 inhibition significantly increased the proliferation, migration and invasion potential of A549 cells (Supplementary Figure S11; *P*<0.05). Taken together, these *in vitro* results suggest that reinforcement of hsa-miR-623 expression significantly inhibits cell proliferation, migration and invasion in lung adenocarcinoma.

### Hsa-miR-623 inhibits xenografts growth and metastasis *in vivo*

Sixty 4-week old male athymic nu/nu mice were divided into six groups (*n*=9–10 per group). The mice received 3 × 10^6^ cells of miR-623-expressing clones and the NC-transfected A549 or PC-9 clone cells, respectively, by subcutaneous injection into the flank. Tumor volumes were measured with calipers every 4 days after injection. The tumors were removed from the killed mice on day 24 after injection. As shown in Figures 4a and b, the mean volumes of the tumors derived from the miR-623-expressing clones were significantly smaller than those derived from the NC-transfected clone cells both in A549 and PC-9 (*P*<0.01). In addition, tumors derived from the miR-623-expressing clone cells (both in A549 and PC-9 cells) grew at significantly slower rates at all time points examined since day 12 after injection relative to the control groups (*P*<0.01; Figures 4c and d).

The preceding *in vitro* studies indicated that miR-623 could suppress the migration and invasion of lung adenocarcinoma cells. Thus, we established an orthotopic tumor nude mice model to evaluate the effect of hsa-miR-623 on lung adenocarcinoma cell distant metastasis *in vivo*. Injection of cancer cells into the thoracic cavity of nude mice closely mimicked orthotopic lung tumor growth. Compared with the control mice groups, mediastinum lymph node metastasis and two lung metastatic nodules were significantly decreased in hsa-miR-623-overexpression mice groups (Figures 4e–g; *P*<0.05). In addition, the number of liver metastasis nodules was also markedly decreased in the miR-623-overexpression group compared with the control group (Figures 4e and h; *P*<0.05). In addition, the ratio of lung metastasis, mediastinum lymph node metastasis and liver metastasis in the hsa-miR-623 overexpression group was markedly lower than those of the controls (Figures 4f–h; *P*<0.05).

### Hsa-miR-623 suppresses lung adenocarcinoma cell growth, migration and invasion by downregulating Ku80 expression

To confirm the involvement of Ku80 in the antitumor effects of hsa-miR-623, we transfected Ku80-expressing lentiviral vector (GV320-Ku80) and empty lentiviral vector (GV320) into A549-miR-623 #1 cells for further experiments. After GV320-Ku80 was introduced into the A549-miR-623 #1 cells, suppression of cell proliferation, clonogenicity, migration and invasion induced by hsa-miR-623 was reversed to a certain extent (Figures 5a–d). Relative to the control group, overexpression of Ku80 in A549-miR-623 #1 cells significantly promoted subcutaneous tumor growth *in vivo* (*P*<0.05; Figures 5e and f). These results suggested that reintroduction of Ku80 partially abrogates miR-623-induced suppression of lung adenocarcinoma growth and metastasis.

The article "Hsa-miR-623 suppresses tumor progression in human lung adenocarcinoma" was retracted in 2019. Reasons: contaminated cell lines or tissues; unreliable results or conclusions.

To further identify the role of Ku80 in lung adenocarcinoma pathogenesis, we examined whether inhibition of Ku80 resulted in repression of lung adenocarcinoma, similar to that observed with miR-623 overexpression. Ku80 siRNA and control siRNA were introduced into NC-transfected A549 cells. We observed that specific knockdown of Ku80 by siRNA could result in the suppression of cell proliferation, clonogenicity, migration and invasion, similar to that seen in A549-miR-623 #1 cells (Figures 5a–d). In the nude mouse model, compared with the control group, intratumor injection of cholesterol-conjugated Ku80 siRNA inhibited Ku80 expression and significantly suppressed subcutaneous tumor growth (*P*<0.05; Figures 5e and f).

Hsa-miR-623 overexpression and Ku80 inhibition produce similar changes, which are restored by Ku80 ectopic expression *in vitro* and *in vivo*. In summary, these data suggest that negative regulation of Ku80 contributed to the antitumor effects of hsa-miR-623 involved in lung adenocarcinoma. Meanwhile, hsa-miR-623 might have additional targets that assist in its tumor suppressive effect, except Ku80.

### Hsa-miR-623 decreases MMP-2/9 expressions and inhibits activation of the ERK/JNK pathway

We examined the levels of several epithelial–mesenchymal transition and adhesion-related molecules, such as E-cadherin, N-cadherin, snail and vimentin, and did not find significant changes (Figure 6a). MMPs are well-documented extracellular membrane-degrading enzymes associated with tumor invasiveness.^26^ We next determined whether hsa-miR-623 overexpression, which led to inhibition of cell invasion, occurred as a result of decreased MMPs levels. MMP-2 and MMP-9 protein levels were measured by using western blot analysis and gelatin zymography. The data showed that hsa-miR-623 resulted in downregulation of MMP-2 and MMP-9 expressions (Figure 6a; *P*<0.01). Consistent with the results, gelatin zymography showed lytic zones at the molecular mass corresponding to MMP-9 and MMP-2. Hsa-miR-623 resulted in decreasing secretion and enzyme activity of MMP-2 and MMP-9 (Figure 6b; *P*<0.05). Because previous studies have shown that the mitogen-activated protein kinase (MAPK) pathway is critical for the activation of MMPs transcription,^27, 28^ we ask if hsa-miR-623 plays a role in regulating the MAPK pathway. We examined the levels of total and phosphorylated(active) forms of MAPK family members (ERK1/2, JNK and P38 MAPK) in A549 cells treated with hsa-miR-623 overexpression. As shown in Figure 6c, hsa-miR-623 overexpression significantly decreased ERK1/2 and JNK activation (*P*<0.01), but not the inactivation of p38 MAPK (*P*>0.05). Meanwhile, hsa-miR-623 inhibition could significantly increase the MMP-2/9 expressions and activate the ERK/JNK pathway (Supplementary Figure S11; *P*<0.05). Immunohistochemical staining study indicated that Ku80, p-ERK, p-JNK, MMP-2 and MMP-9 expressions were also decreased in the tumor tissues derived from the miR-623-expressing cells compared with those in the tumors from the NC-transfected A549 cells (Figure 6d; *P*<0.01; Suplementary Material and Supplementary Figure S7). Western blot analysis also showed that expression levels of MMP-2, MMP-9, p-ERK and p-JNK in lung adenocarcinoma tissues were increased compared with those in normal tissues (Supplementary Figure S5).The alteration patterns of these protein expressions in xenograft tumor tissues and human tissues were consistent with those protein expressions identified *in vitro* in miR-623-expressing cells and NC-transfected cells.

The article "Hsa-miR-623 suppresses tumor progression in human lung adenocarcinoma" was retracted in 2019. Reasons: contaminated cell lines or tissues; unreliable results or conclusions.

### The inhibitory effect of hsa-miR-623 on cell invasion by targeting Ku80 may be through ERK/JNK inactivation mediating MMP-2/9 downregulation

Next, we asked whether ERK/JNK mediates hsa-miR-623 suppression of MMP-2/9 expression. As shown in Figures 7a and b, hsa-miR-623 overexpression or Ku80 knockdown significantly decreased the MMP-2/9 expression levels, and inhibited the ERK and JNK activation. The ERK inhibitor (PD98059) or JNK inhibitor (SP600125) was used to inhibit ERK or JNK activation. Basal MMP-2 and MMP-9 production and invasion ability were inhibited by treatment of A549 cells with PD98059 or SP600125, similar to that seen in A549 cells transfected with miR-623 mimics, while the Ku80 expression level remained unchanged in the A549-NC cells treated with PD98059 or SP600125. Furthermore, hsa-miR-623 inhibition or Ku80 overexpression induced MMP-2/9 production and increased invasion ability, as well as activated the ERK and JNK pathway in HBE cells (Figures 7c and d). The increased invasive ability induced by hsa-miR-623 inhibition in HBE cells was reversed by targeted inhibition using PD98059 or SP600125 (Figures 7c and d). While, hsa-miR-623 inhibition increased Ku80 expression level remains unchanged when the HBE cells treated with PD98059 or SP600125 (Figure 7c). It had also been validated that hsa-miR-623 expression did not show any significant change when receiving JNK inhibitors both in A549 and PC-9 cells (Supplementary Figure S10; *P*>0.05).

The article "Hsa-miR-623 suppresses tumor progression in human lung adenocarcinoma" was retracted in 2019. Reasons: contaminated cell lines or tissues; unreliable results or conclusions.

Therefore, hsa-miR-623 may suppress lung adenocarcinoma cells invasion by targeting Ku80 through ERK/JNK inactivation mediated downregulation of MMP-2/9.

## Discussion

Many studies have shown that miRNAs can function as oncogenes or tumor suppressors by post-transcriptionally inhibiting numerous target gene expressions in lung cancer.^16^ We successfully identified two miRNAs (hsa-miR-526b and hsa-miR-623) that could significantly inhibit Ku80 expression in A549 cells in our previous study.^10^ Our previous study had explored the function of hsa-miR-526b in NSCLC,^10^ so we chose to investigate the role of hsa-miR-623 in this paper. The present data demonstrated that hsa-miR-623 directly bound to the 3′-UTR of Ku80 mRNA and markedly inhibited Ku80 expression. Hsa-miR-623 was found to be frequently downregulated in lung adenocarcinoma tissues when compared with adjacent non-cancerous tissues, and it showed an inverse significant correlation with Ku80 expression. Clinicopathological correlation analysis showed that hsa-miR-623 expression was significantly correlated with tumor differentiation, smoking history, lymphatic metastasis and elevated serum CEA level in patients with lung adenocarcinoma, which was similar to the results found in the study of Ku80. Further study indicated that hsa-miR-623 significantly suppressed lung cancer cell proliferation, migration and invasion *in vitro*. Hsa-miR-623 was shown to significantly inhibit tumor growth and metastasis in nude mouse model. Taken together, these data suggested that hsa-miR-623 functioned as a tumor suppressor in lung adenocarcinoma. To the best of our knowledge, this is the first attempt to illuminate the expression pattern of hsa-miR-623 and its role in lung adenocarcinoma using both *in vitro* and *in vivo* models.

Further studies were performed to illustrate the molecular mechanisms of tumor metastasis inhibition of hsa-miR-623 in lung adenocarcinoma. Our study showed that an inverse correlation was observed between hsa-miR-623 and Ku80 expressions. In addition, silencing of Ku80 by RNAi inhibited tumor metastasis of lung cancer cells in a manner resembling that of hsa-miR-623 overexpression. This result was consistent with a recent study showing that a novel antibody (7B7) directed against the Ku70/Ku80 heterodimer blocks invasion in pancreatic and lung cancer cells.^12^ Moreover, restoration of Ku80 could partially reverse the tumor metastasis inhibition induced by hsa-miR-623 *in vitro*. Thus, downregulation of Ku80 may, at least partially, explain the tumor metastasis inhibition of hsa-miR-623 in lung adenocarcinoma. Tumor invasion is a phenomenon that requires decreased adhesion, increased motility and proteolysis.^14^ We examined the levels of several epithelial–mesenchymal transition and adhesion-related molecules, such as E-cadherin, N-cadherin, snail and vimentin, and did not find significant changes. Our data demonstrated that hsa-miR-623 inhibited lung adenocarcinoma cell invasion through decreasing expression levels of MMP-2 and MMP-9. Metalloproteinases (MMPs) are largely implicated in promoting angiogenesis, tumor invasion and tumor metastasis.^29^ Above all, MMP-2 and MMP-9 have been suggested to be critical for the invasive and metastatic potential in lung carcinoma. The upregulation of MMP-2 and MMP-9 is associated with poor prognosis in patients with lung cancer.^30, 31^ MMP-2 and MMP-9 expression levels are reported to be regulated by numerous oncogene and tumor suppressor pathways.^32^ MAPK is one of the signaling pathways known to mediate metastasis via transmission of extracellular stimuli into the nucleus that activate the serine/threonine kinases.^33^ MAPK pathways involving JNK, p38 and ERK signaling have been reported to upregulate the expression of MMPs.^34, 35^ Regulation of metastasis by MAPK is mainly via controlling the cells' expression of MMPs enzymes by decreasing the nuclear levels of NF-*κ*B, c-Fos or c-Jun.^33, 36^ The present study shows that hsa-miR-623 overexpression leads to significantly reduction in the expressions of Ku80, p-ERK, p-JNK, MMP-2/9 and reduces lung adenocarcinoma cell invasion. Moreover, it is established that hsa-miR-623 inhibition increases Ku80 expression, leads to ERK/JNK family activation, and increases tumor invasion. In keeping with this observation, inhibition of ERK or JNK signaling blocks invasion and reduces MMP-2/9 expression in lung adenocarcinoma cells. Furthermore, hsa-miR-623 inhibition or Ku80 overexpression induced MMP-2/9 production and increased invasion ability, as well as activated the ERK and JNK pathway in HBE cells. The increased invasive ability induced by hsa-miR-623 inhibition in HBE cells was reversed by targeted inhibition using PD98059 or SP600125. These results suggested that the hsa-miR-623 may inhibit cell invasion by targeting Ku80 through inactivating ERK/JNK pathway mediated downregulation of MMP-2/9. Consistent with our results, Xiao *et al.*^37^ reported that Ku80 knockdown suppressed lung cancer growth, resulting in an inactivation of ERK/MAPK pathway. Yang *et al.*^38^ found that 3,5,4′-trimethoxy-trans-stilbene inhibited invasion of human lung adenocarcinoma cells by suppressing the MAPK pathway and decreasing MMP-2 expression. The butanol fraction of guava leaf extract suppressed MMP-2 and MMP-9 expression and activity through the suppression of the ERK1/2 signaling pathway, resulting in suppression of lung cancer cell invasion and metastasis.^39^ Indeed, a single miRNA has been thought to target multiple mRNAs and regulate gene expression.^40^ Therefore, there may be other molecules or signaling pathways which are also targeted by hsa-miR-623, and some of them may be still unknown in lung adenocarcinoma. This presumption may guide future studies to determine the functions of hsa-miR-623 in lung adenocarcinoma carcinogenesis and progression.

The article "Hsa-miR-623 suppresses tumor progression in human lung adenocarcinoma" was retracted in 2019. Reasons: contaminated cell lines or tissues; unreliable results or conclusions.

Taken together, our results demonstrate that hsa-miR-623 directly targets Ku80, which inhibits tumor migration and invasion by downregulating MMP-2/9 through ERK/JNK pathway. Moreover, overexpression of hsa-miR-623 or knockdown of Ku80 significantly suppresses the lung adenocarcinoma progression *in vitro* and *in vivo*. Our studies provide a rationale for the development of hsa-miR-623 or Ku80 as a potential therapeutic target against lung adenocarcinoma.

## Materials and Methods

### Antibodies and reagents

Ku80 siRNA used for *in vitro* transfection and *in vivo* cholesterol-conjugated Ku80 siRNA delivery, hsa-miR-623 mimics and inhibitors and their respective NCs were from Ribobio Company (Guangzhou, China). The hsa-miR623-expressing plasmid, GV252-miR-623, the Ku80-expressing lentiviral vector, GV320-Ku80, and their corresponding control vectors were purchased from Genechem (Shanghai, China). Anti-Ku80 (Ab-2), ERK1/2 (4695), Phospho-ERK1/2(9106), JNK(3708), Phospho-JNK(4668), P38(8690), Phospho-P38(9215), MMP-2(2C1), MMP-9(2C3), Snail(C15D3), Vimentim(D21H3), N-cadherin(24E10), E-cadherin (24E10) and *β*-actin (D6A8) antibodies were purchased from Cell Signaling Technology (Beverly, MA, USA). ERK inhibitor (PD98059) and JNK inhibitor (SP600125) were purchased from Sigma (St. Louis, MO, USA).

### Patients and specimens

Eighty-nine pairs of human lung adenocarcinoma tissues and their corresponding adjacent lung samples were obtained from patients who underwent lung resection surgery at the Thoracic Surgery Center of Tongji Hospital affiliated with Huazhong University of Science and Technology between 2007 and 2011. Lung adenocarcinoma tissues were confirmed pathologically, and all specimens were stored at −80 °C until used for analysis. Clinicopathologic histories for these patients including age, gender, differentiation, smoking history, pathological pattern, lymphatic metastasis, tumor diameter, serum CEA level and tumor staging are shown in Table 1. Lung cancer was staged according to the tumor-node-metastasis (TNM) staging system of the Union for International Cancer Control (UICC).^41^ All the patients underwent radical surgery. Patients with preoperative chemotherapy or radiotherapy treatment or with evidence of other malignancies were excluded. No patients received gene-targeted therapy during the follow-up period. Overall survival was defined as the time from the diagnosis until time of death from any cause. Cases lost to failure to follow-up and deaths caused by conditions other than lung cancer were regarded as censored data in the survival analysis. This study was approved by the medical ethics committee of Tongji Hospital and informed consent was obtained from all patients.

The article "Hsa-miR-623 suppresses tumor progression in human lung adenocarcinoma" was retracted in 2019. Reasons: contaminated cell lines or tissues; unreliable results or conclusions.

### Western blot analysis

The cell cultures and tissues were lysed in ice-cold RIPA lysis buffer (50 mM Tris-HCl, 1% NP40, 0.1% SDS, 0.5% sodium deoxycholate, 0.02% sodium azide, 150 mM NaCl at pH 8.0) containing protease inhibitor cocktail (Roche, Basel, Switzerland). After the protein concentration was determined using a BCA Kit (Pierce, Rockford, IL, USA), 60 *μ*g of proteins were separated on pre-casted 10% SDS-polyacrylamide gels and then electrotransferred onto PVDF membranes (Millipore, Billerica, MA, USA) in transfer buffer. The blots were blocked in 5% non-fat milk for 2 h and incubated overnight at 4 °C with primary antibodies (1 : 1000 dilution). The blots were then incubated with horseradish peroxidase-conjugated secondary antibody at 1 : 5000 dilution for 1 h at 37°C. The signals were visualized using the enhanced chemiluminescence system (Pierce, USA). Protein expression was quantified by densitometry and normalized to *β*-actin expression using Alpha View software.

### Immunohistochemical staining

Antigen retrieval in the tissue sections was performed in boiling citrate buffer for 15 min. Peroxide blocking was conducted with 0.3% peroxide in absolute methanol. After the slides had been incubated overnight with primary antibodies (1 : 200 dilution) at 4 °C and washed twice with phosphate-buffered saline (PBS), they were then incubated with secondary antibody (Dako, Glostrup, Denmark) at 37 °C for 30 min. After washing, the color reaction was developed with DAB work solution (Dako). The immunostaining results were assessed and scored independently by two pathologists as described previously.^42^

The article "Hsa-miR-623 suppresses tumor progression in human lung adenocarcinoma" was retracted in 2019. Reasons: contaminated cell lines or tissues; unreliable results or conclusions.

### RNA isolation and qRT-PCR assays

Total RNAs from both fresh tissues and cell lines were extracted with Trizol reagent (Invitrogen, Grand Island, NY, USA). MiRNAs from formalin-fixed and paraffin-embedded samples were extracted by using the RNeasy FFPE Kit (Qiagen, Hilden, Germany). The first strand of complementary DNA was generated with a reverse-transcription system kit (Toyobo, Osaka, Japan). Stem–loop reverse transcription for mature hsa-miR-623 and U6 RNA was obtained from Ribobio Company. U6 RNA was used as the miRNA internal control and normalizer for miRNA qRT-PCR experiments (Ct values of U6 in tissue samples were shown in Supplementary Table S1).The qRT-PCR was performed with a standard SYBR-Green PCR kit (Toyobo) according to a Step One system protocol (Applied Biosystems, Foster City, CA, USA). The qRT-PCR reactions were performed in triplicate. Data analysis was performed using the 2^−ΔΔCt^ method.

### Cell culture and transfection

The human lung adenocarcinoma cell lines (A549 and PC-9) and HBE cell lines were all obtained from the Center for Type Culture Collection of China and maintained in DMEM (Gibco, Waltham, MA, USA). Cells were supplemented with 10% fetal bovine serum (Gibco,Waltham, MA, USA). The A549 and PC-9 cells were transiently transfected with the RNAs or vector by using Lipofectamine 2000 (Invitrogen) following the manufacturer's protocol. The A549 cells were infected by GV320-Ku80 lentiviral vector and GV320 lentiviral vector according to the manufacturer's protocol. At the indicated time points, the cells were harvested for use in the western blot analysis and cell proliferation assays. For stable transfections, 5 × 10^5^ cells per well were seeded in a six-well plate for 24 h. Plasmid was delivered into the cells using Lipofectamine 2000 following the manufacturer's protocol. After culturing in medium containing 400 *μ*g/ml of G418 (Calbiochem, Darmstadt, Germany) for 3 weeks, the individual clones were isolated. The positive cell clones that stably expressed hsa-miR-623 were then identified using qRT-PCR. The clones stably expressing hsa-miR-623 were maintained in medium containing 250 *μ*g/ml of G418 for further experiments.

### Luciferase reporter assay

To verify the precise target of miRNAs, the Dual-Luciferase Reporter Assay System (Promega, Madison, WI, USA) was used. Briefly, 5 × 10^5^ lung adenocarcinoma cells were seeded in 24-well plates. After 24 h, the luciferase reporter plasmids (pLUC, pLUC-wt-Ku80 and pLUC-mutant-Ku80) were co-transfected with GV252-miR623 (miR-623), or GV252 (miR-NC) using Lipofectamine 2000 (Invitrogen). Firefly and renilla luciferase activities were measured at 48 h post-transfection using the Dual-Glo Luciferase Assay System (Promega). Firefly luciferase was normalized to renilla luciferase activity. All experiments were performed three times.

The article "Hsa-miR-623 suppresses tumor progression in human lung adenocarcinoma" was retracted in 2019. Reasons: contaminated cell lines or tissues; unreliable results or conclusions.

### Cell proliferation assay

Cells (5000 per well) were plated in 96-well plates and incubated at 37 °C. Cell proliferation was assessed at indicated times after transfection using the Cell Counting Kit-8 (Dojindo, Kumamoto, Japan) according to the manufacturer's instruction. Each assay was repeated independently three times.

### Analysis of clonogenicity *in vitro*

For plate colony formation analysis, 100 viable lung adenocarcinoma cells were placed in 24-well plates 24 h after transfection and were maintained in complete medium for 2 weeks. Colonies were fixed with methanol and stained with 0.1% crystal violet in 20% methanol. Soft agar colony formation assay was performed according to the methods described previously. Briefly, 1000 cells were equally divided into four wells in a 24-well plate in medium containing 0.3% noble agar and grown for 14–21 days. The number of colonies was determined by direct counting using an inverted microscope (Nikon, Tokyo, Japan).

### Cell migration and invasion assay

A cell invasion and migration assay was performed using a 24-well transwell chamber with a pore size of 8 mm (Costar, Corning, NY, USA), and the inserts were coated with or without 20 *μ*l of 1 : 4 dilution Matrigel (BD Bioscience, San Jose, CA, USA). Cells were trypsinized, transferred to the upper chamber in 100 *μ*l of serum-free medium containing 3 × 10^5^ cells and incubated for 18–24 h. Medium supplemented with 10% fetal bovine serum was added to the lower chamber as the chemoattractant. Then, the non-invading cells on the upper membrane surface were removed with a cotton tip, and the cells that passed through the filter were fixed in 4% paraformaldehyde and stained with methyl violet. The experiments were performed in triplicate.

### Gelatin zymography assay

Gelatin zymography was used to analyze MMP-2 and MMP-9 in the supernatant of cultured cells. Gelatin zymography assay was performed according to the methods described previously.^26^

### Animal studies

BALB/c athymic nude mice (male, 4-week-old and 16–20 g) were purchased from Hubei Research Center of Laboratory Animal (Wuhan, China) and bred at pathogen-free conditions in Animal Center of Tongji Medical College. The hsa-miR-623-expressing and NC-transfected clone cells were harvested and resuspended to 3 × 10^7^ cells/ml in PBS. We injected 3 × 10^6^ cells in a total volume of 100 *μ*l subcutaneously into the right flank of athymic nude mice (*n*=9–10/clone). For the rescue experiment, the mice were randomly divided into six groups (*n*=4/group). The initial four groups of mice, A549-NC (group 1), A549-miR-623#1 (group 2), A549-miR-623#1 transfected with GV320 (group 3) and A549-miR-623#1 transfected with GV320-Ku80 (group 4), received subcutaneous injections of cells into the flank. Two other groups received injections of A549-NC cells. Eight days were allowed for tumor development. After this period, Ku80 siRNA or control siRNA was directly injected into the implanted tumor at the dose of 1nmol (in 20 *μ*l PBS) per mouse every 4 days for a total of five times in each group. Tumor size was monitored every 4 days and measured using a caliper. The tumor volume was calculated by the formula *V* (cm^3^)=*L* × *W*^2^/2, where *L* represents the longest dimension and *W* the shortest dimension of the tumor. Twenty-four days after injection, the mice were killed and their tumors removed. Tumor tissue fragments were fixed in 10% formalin and stored in −80 °C at the same time. Expressions of Ku80, MMP-2, MMP-9, p-JNK and p-ERK in xenograft tumor tissues were detected by immunohistochemistry.

The article "Hsa-miR-623 suppresses tumor progression in human lung adenocarcinoma" was retracted in 2019. Reasons: contaminated cell lines or tissues; unreliable results or conclusions.

The A549-NC and A549-miR-623#1 clone cells (5 × 10^5^ cells in 50 *μ*l of PBS containing 25 ng of Matrigel; BD) were injected into the left pleural cavities of 4-week-old male athymic nude mice (*n*=8 per group) to construct the orthotopic model according to the methods described previously. The mice were killed by overexposure to CO_2_ 30 days after implantation, at which time the two lungs (including heart and mediastinum tissues) and liver were removed and fixed in 10% formalin. Further, in-depth quantitative analysis of tumor burden was assessed on the lungs, mediastinum or liver, which was fixed and cut sagittally into four parts, paraffin-embedded, sectioned and stained for H&E. Slides were scanned at × 20 using an Ariol SL-50scanner (Leica Biosystems, Nussloch, Germany). The lung, mediastinum and liver nodules were counted by microscopic examination. Ariol software was used to quantify the size and number of tumors per section.

### Statistical analysis

Data were imaged with GraphPad Prism 5 software (GraphPad Software, La Jolla, CA, USA). All results represent the average from triplicate experiments are expressed as the mean±standard deviation. The associations between categorical variables were assessed using the chi-square test or the Fisher exact test. Overall survival was calculated using the Kaplan–Meier method and log-rank tests. Analysis of variance (ANOVA) was performed to determine statistically significant differences between the groups. A value of *P*<0.05 was considered statistically significant.

## Figures and Tables

**Figure 1:** Hsa-miR-623 directly targets Ku80 in lung adenocarcinoma cells. (**a**) Predicted consequential pairing of wild type or mutant 3′-UTR of Ku80 mRNA and hsa-miR-623 by Targetscan. (**b**) Luciferase assays in A549 and PC-9 cells. PLUC, pLUC-wtKu80 and pLUC-mutKu80 vectors were co-transfected with pre-miR-623 or pre-miR-NC. Relative suppression of luciferase expression was standardized to *β*-gal signal. Luciferase activity in the pLUC-wtKu80 group displayed a significant decrease following ectopic expression of hsa-miR-623. (**c** and **d**) Ku80 protein was measured by western blot analysis 48 h after transfection. (**c**) Ku80 protein was downregulated in A549 and PC-9 cells transfected with hsa-miR-623 mimics. (**d**) Ku80 protein was upregulated in A549 and PC-9 cells with hsa-miR-623 inhibitor. *P<0.05

**Figure 2:** Hsa-miR-623 is downregulated in lung adenocarcinoma tissues and its downregulation is inversely correlated with Ku80 overexpression. (**a**) Downregulation of hsa-miR-623 in lung adenocarcinoma tissues compared with adjacent lung tissues (measured by TaqMan qRT-PCR, *P*<0.001 compared with controls). (**b**) Kaplan–Meier analysis of overall survival in all lung adenocarcinoma patients according to hsa-miR-623 expression level. (**c**) Quantitative analysis of Ku80 expression in 89 cases of paired lung adenocarcinoma tissues and their corresponding adjacent lung tissues by western blot analysis. The *P*-value (*P*=0.0021) corresponds to the comparison of Ku80 expression between the lung adenocarcinoma tissues and corresponding adjacent lung tissues. (**d**) Downregulation of hsa-miR-623 is inversely correlated with Ku80 upregulation (*R*=−0.631, *P*<0.0001, Pearson's correlation)

**Figure 3:** Hsa-miR-623 suppresses growth, migration and invasion of lung adenocarcinoma cells *in vitro*. (**a**) Relative expression of hsa-miR-623 detected by TaqMan qRT-PCR in two lung adenocarcinoma cell lines stably transfected with hsa-miR-623 or hsa-miR-NC. (**b**) Hsa-miR-623 overexpression significantly suppressed the proliferation of A549 and PC-9 cells by using CCK8 assay. (**c**) Histograms indicated that hsa-miR-623 can markedly inhibit the plate colony formation in A549 and PC-9 cells. (**d**) Histograms showed that hsa-miR-623 significantly suppressed anchorage-independent cell growth in A549 and PC-9 cells. (**e**) and (**f**) represent the results of cell migration and invasion in transwell assays with or without Matrigel. (**g**) and (**h**) Histograms indicate the relative number of migratory or invasive cells across a membrane with 8 mm pores with or without Matrigel, respectively. The results are representative of three independent experiments. Data are given as means±S.D., *P<0.05 compared with controls

**Figure 4:** The suppressive role of hsa-miR-623 on xenografts growth in *vivo* and metastasis in orthotopic lung cancer nude mice model. (**a** and **b**) The subcutaneous tumors derived from the hsa-miR-623-overexpressing clones were smaller than those from the NC-transfected clones in A549 and PC-9 cells. (**c** and **d**) Tumor growth curves showed that tumors derived from the hsa-miR-623-overexpressing A549 or PC-9 cells grew significantly slower than those from the control cells at all time points past 12 days after injection. (**e**) Representative photographs of mouse two lungs, mediastinum and liver, as well as images of the histological inspection of mouse two lungs, mediastinum and liver for the presence of microscopic lesions at 4 weeks after thoracic injection with A549 cells stably expressing miR-623 or the negative control lentiviral vector. (**f**–**h**) Quantification of microscopic nodules and incidence of metastasis in the mediastinum, contralateral lung and liver of each group, respectively. The results shown represent the mean±S.D. of triplicate experiments. *P<0.05

**Figure 5:** Hsa-miR-623 suppresses lung adenocarcinoma cell growth, migration and invasion by downregulating Ku80 expression. (**a**) Cell proliferation detected in different cell groups at 0, 1, 3 and 5 days after transfection. (**b**) Histogram illustrated the relative colony numbers per field of indicated cell groups. (**c** and **d**) Histograms of migratory (**c**) and invasive (**d**) cell numbers per field of the indicated cell groups. (**e**) Subcutaneous tumors derived from indicated cell groups (*n*=4 each). (**f**) Tumor growth curves demonstrating that transfection of GV320-Ku80 in A549-miR-623 #1 cells significantly promoted subcutaneous tumor growth, while intratumoral injection of cholesterol-conjugated Ku80 siRNA significantly suppressed subcutaneous tumor growth compared with control groups. The mean and S.D. for tumor volumes were determined for each group. NS, *P*>0.05; *P<0.05

**Figure 6:** Hsa-miR-623 decreases MMP-2/9 expression and inhibits activation of the ERK/JNK pathway. (**a**) Western blot analysis showing the expressions of E-cadherin, N-cadherin, Vimentin, Snail, MMP-2 and MMP-9 in A549 and PC-9 cells stably transfected with the miR-623-expressing vector or empty vector. *β*-Actin was used as a loading control. (**b**) Conditioned medium from each group were collected and analyzed for MMP-2 and MMP-9 expression by gelatin zymography. (**c**) Western blot analysis showing the expression levels of Ku80, MMP-2, MMP-9, as well as activities of ERK1/2, p38 and JNK for total and phosphorylated forms. (**d**) Immunohistochemistry showing the expression status of Ku80, p-JNK, p-ERK, MMP-2 and MMP-9 in the xenograft tumor tissues. Data are given as means±S.D. *P<0.05

**Figure 7:** Hsa-miR-623 may inhibit cell invasion by MMP-2/9 downregulation through ERK/JNK pathway. (**a**) A549 cells were transfected with negative control RNA, hsa-miR-623 mimics or Ku80 siRNA, followed by JNK inhibitor (SP600125) and the ERK inhibitor (PD98059) treatment. Whole-cell lysates were analyzed for the protein levels of Ku80, MMP-2, MMP-9, p-JNK, p-ERK, t-JNK and t-ERK. (**b**) Cell invasion was evaluated using Matrigel-coated filters for 24 h after miRNA mimics treatment or 2 h after inhibitors treatment. (**c**) HBE cells were transfected with negative control RNA, hsa-miR-623 inhibitor or Ku80-overexpressed vector, followed by JNK inhibitor (SP600125) and the ERK inhibitor (PD98059) treatment. Expression levels of Ku80, MMP-2, MMP-9, p-JNK, p-ERK, t-JNK and t-ERK were determined by western blot analysis. (**d**) Matrigel cell invasion was evaluated. Data are given as means±S.D. invaded cells per field. *P<0.05

**Table 1:** Correlation between hsa-miR-623 downregulation and clincopathological parameters in the patients with lung adenocarcinoma

**Variables**	**Total cases (*****n*****=89)**	**miR-623 expression level**		***P*-value**^a^
		**Downregulated (*****n*****=72)**	**Intact (*****n*****=17)**	
*Age (years)*				0.344
≤50	56	47	9	
>50	33	25	8	
				
*Gender*				0.610
Male	52	43	9	
Female	37	29	8	
				
*Differentiation*				0.006^b^
Low	43	39	4	
Moderate	28	23	5	
High	18	10	8	
				
*Smoking history*				0.513
Never	46	36	10	
Ever	43	36	7	
				
*Lymphatic metastasis*				0.011^b^
Yes	21	13	8	
No	68	59	9	
				
*Tumor diameter (mm)*				0.0498^b^
≤50	63	50	13	
>50	26	22	4	
				
*CEA (ng/ml)*				0.001^b^
≤5	47	32	15	
>5	42	40	2	
				
*Staging*				0.431
I–II	39	33	6	
III–IV	50	39	11	

a Chi-square test or the Fisher exact test.

b Statistically significant (*P*<0.05)

The article "Hsa-miR-623 suppresses tumor progression in human lung adenocarcinoma" was retracted in 2019. Reasons: contaminated cell lines or tissues; unreliable results or conclusions.

## Abbreviations

MAPK: mitogen-activated protein kinases
t-ERK: total-extracellular signal-regulated kinases
t-JNK: total-c-Jun N-terminal kinases
p-ERK: phosphor-extracellular signal-regulated kinases
p-JNK: phosphor-c-Jun N-terminal kinases
MMP: matrix metalloproteinase
3′-UTR: 3′-untranslated regions
NSCLC: non-small cell lung cancer
DSBs: DNA double-strand breaks
miRNA: microRNA
hsa-miR: Homo sapiens miRNA
siRNA: small interfering RNA
CEA: carcinoembryonic antigen
HBE: human bronchial epithelial cells
qRT-PCR: quantitative real-time polymerase chain reaction
